# Differential Expression Profiling of Spleen MicroRNAs in Response to Two Distinct Type II Interferons in *Tetraodon nigroviridis*

**DOI:** 10.1371/journal.pone.0096336

**Published:** 2014-05-06

**Authors:** Shibai Yi, Danqi Lu, Wan Peng, Ting Wang, Yong Zhang, Haoran Lin

**Affiliations:** State Key Laboratory of Biocontrol, Institute of Aquatic Economic Animals and Guangdong Provincial Key Laboratory for Aquatic Economic Animals, College of Life Sciences, Sun Yat-Sen (Zhongshan) University, Guangzhou, PR China; Friedrich-Loeffler.Institut, Germany

## Abstract

MicroRNAs are endogenous, small non-coding RNAs approximately 18–26 nucleotides in length that regulate target gene expression at the post-transcription level. Interferon-γ (IFN-γ) is a Th1 cytokine that is involved in both the innate and adaptive immune responses. We previously identified two IFN-γ genes in green-spotted puffer fish (*Tetraodon nigroviridis*). To determine whether miRNAs participate in IFN-γ-related immune responses, *T. nigroviridis* spleen cells were treated with recombinant IFN-γ isoforms, and a Solexa high-throughput sequencing method was used to identify miRNAs. In total, 1,556, 1,538 and 1,573 miRNAs were found in the three samples, and differentially expressed miRNAs were determined. In total, 398 miRNAs were differentially expressed after rIFN-γ1 treatment, and 438 miRNAs were differentially expressed after rIFN-γ2 treatment; additionally, 403 miRNAs were differentially expressed between the treatment groups. Ten differentially expressed miRNAs were chosen for validation using qRT-PCR. Target genes for the differentially expressed miRNAs were predicted, and GO and KEGG analyses were performed. This study provides basic knowledge regarding fish IFN-γ-induced miRNAs and offers clues for further studies into the mechanisms underlying fish IFN-γ-mediated immune responses.

## Introduction

MicroRNAs (miRNAs) are small non-coding RNAs that regulate target messenger RNA (mRNA) expression by binding to mRNA 3' untranslated regions (3' UTR), resulting in mRNA cleavage or translational repression through the RNA-induced silencing complex (RISC) [1]. MiRNAs play an important role in many biological processes, such as development [2], [3], cell proliferation, differentiation and death [4], [5], [6], [7], tumorigenesis [8], [9], and inflammation [10], [11], in addition to several diseases [12], [13]. In recent years, with the development of high-throughput sequencing technologies, miRNAs have been increasingly identified in teleosts such as Japanese flounder (*Paralichthys olivaceus*) [14], Atlantic salmon (*Salmo salar*) [15], Atlantic halibut (*Hippoglossus hippoglossus*) [16], [17], and channel catfish (*Ictalurus punctatus*) [18]. Several miRNA expression studies have been performed in zebrafish, including miRNA profiling during development [19], miRNA profiling in response to LPS and bacterial infection [20], and miRNA profiling induced by PFOS [21].

Interferon (IFN)-γ, the only type II IFN [22], regulates immune processes, including antigen presentation, antiviral response, macrophage activation, and apoptosis [23], by binding to the IFN-γ receptor (IFNGR) [24]. IFN-γ ligand-receptor binding results in activation of Janus tyrosine kinase (Jak)1 [25], followed by phosphorylation of the signal transducer and activator of transcription (Stat)1. The Stat1-Stat1 homodimer binds to GAS (interferon-gamma activated sequence) elements in the promoters of IFN-γ-regulated genes and leads to gene regulation [26]. Stat3 and Stat5 can also be activated by IFN-γ in certain cell types [27], [28]. In teleosts, IFN-γ was first identified in Fugu (*Takifugu rubripes*) in 2004 [29]. Fish IFN-γ induces typical IFN-γ-induced genes, including the major histocompatibility complex (MHC) class II and Stat1, and also primes macrophages and enhances respiratory bursting, suggesting that IFN-γ has similar functions in fish and mammals [30], [31], [32]. In contrast to the single copy of the IFN-γ gene that exists in mammalian genomes, two copies of the IFN-γ gene were found in the zebrafish and fugu genomes in 2006; these genes were named IFN-γ1 and IFN-γ2 [33]. The IFN-γ2 gene has proven to be an orthologue of mammalian IFN-γ, whereas IFN-γ1 shares low identity with other species and appears to be fish-specific [34]. Two IFN-γ genes were also found in the channel catfish (*I. punctatus*) [35], common carp (*Cyprinus carpio* L.) [36], goldfish (*Carassius aurutus* L.) [37], and ginbuna crucian carp (*Carassius auratus langsdorfii*) [38]. Both isoforms are members of the type II interferon family and contain IFN-γ signature motifs [30], [33], but the fish-specific IFN-γ1 does not contain the C-terminal nuclear translocation signal (NLS) motif required for IFN-γ activity [35], [39]. Previous studies showed that fish IFN-γ1 and IFN-γ2 exhibited different expression patterns [33], [39] and distinct preferences for different receptors [38], [40], but both induced typical IFN-γ target genes [41], indicating that the two type II IFNs may have separate functions [40], [41]. However, the functional differentiation of the two isoforms and how they differentially regulate downstream genes are still not clear. Because the involvement of miRNAs in the regulation of immune response has been extensively demonstrated [42], [43], it is possible that miRNAs might be involved in fine-tuning the functions of the two type II IFN isoforms.

MiRNAs have been well studied in mammalian inflammation and tumors. Because of the importance of IFN-γ in the immune system, increasing attention has been paid to the miRNA network after IFN-γ stimulation, and several miRNAs have already been reported to act on mammalian IFN-γ. The miR-29 family directly targets IFN-γ [44], and IFN-γ-induced Stat1 can up-regulate miR-29 expression [45]; in cancer cells, miR-145 directly targets Stat1 and c-Myc [46], [47], and miR-378 targets the IFN-γ receptor 1, IFNGR1, to suppress bovine luteal cell apoptosis [48]. However, no study has focused on the miRNA expression profile in response to teleostean IFN-γ stimulation, and comparing the differential expression patterns would provide valuable insight into the separate functions of the two type II interferon isoforms in fish.

The green-spotted puffer fish (*Tetraodon nigroviridis*) has the smallest known vertebrate genome. Little information regarding *T. nigroviridis* miRNAs can be found in the miRBase, and until now, no studies have evaluated *T. nigroviridis* miRNAs and *T. nigroviridis* IFN-γ. We previously identified two IFN-γ genes in the *T. nigroviridis* genome, IFN-γ1 (GenBank accession NO. KJ524454) and IFN-γ2 (KJ524455). Recombinant IFN-γ1 (rIFN-γ1) and IFN-γ2 (rIFN-γ2) from *T. nigroviridis* were produced in *Escherichia coli* using a pET expression vector, as previously described [49], and binding of the recombinant proteins to their receptors was confirmed using ligand binding analysis [49]. In this study, primary cells from the *T. nigroviridis* spleen were treated with rIFN-γ1 and rIFN-γ2. An Illumina deep-sequencing method was performed, and the differential expression of miRNAs was analyzed. These findings will help to determine the roles that miRNA play in regulating IFN-γ-mediated immune responses.

## Materials and Methods

### Ethics statement

All animal experiments were conducted in accordance with the guidelines and approval of the Animal Research and Ethics Committees of Sun Yat-Sen University. All efforts were made to minimize suffering.

### Experiment animals

Green-spotted puffer fish were purchased from the local market and raised for at least one week prior to the experiment. The fish were kept in 28°C circulating water and fed daily. Upon initiation of the experiment, the fish were anesthetized with 1% tricaine methanesulfonate (MS-222), and their spleens were removed and immediately placed in tissue culture medium (RPMI-1640 culture medium supplemented with 10% fetal bovine serum, 2 mM L-glutamine, and 1% penicillin/streptomycin).

### Sample collection and RNA isolation

Primary spleen cells from *T. nigroviridis* were obtained as previously described, with minor modifications [50]. Briefly, tissue culture medium (TCM) was prepared from RPMI-1640 medium (Life Technologies, Gaithersburg, MD, USA) by adding 10% fetal bovine serum (Life Technologies), 2 mM L-glutamine (Sigma, St. Louis, MO, USA), and 1% penicillin/streptomycin (Sigma). Six fish were used in this study; their spleens were removed and immediately kept in TCM. The spleens were then ground into pieces and filtered through a 70- µm cell strainer (BD Falcon, Bedford, MA, USA). The obtained cells were washed and centrifuged with TCM twice, then divided into three groups (Sp-con, Sp-γ1, and Sp-γ2). The cells were then plated in a 6-well plate and incubated at 27°C under 5% CO_2_ for 6 hours before rIFN-γ stimulation. Two IFN-γ genes were previously identified in the *T. nigroviridis* genome and were named IFN-γ1 (GenBank accession NO. KJ524454) and IFN-γ2 (KJ524455). Recombinant IFN-γ1 (rIFN-γ1) and IFN-γ2 (rIFN-γ2) from *T. nigroviridis* was produced as previously described [49]; rIFN-γ1 and rIFN-γ2 proteins at a final concentration of 10 ng/mL were added to the culture medium, and the control group (Sp-con) was treated with TCM. The cells were collected 12 hours after rIFN-γ stimulation, and Trizol (Life Technologies) reagent was immediately added to prevent RNA degradation. Total RNA was extracted using Trizol reagent according to the manufacturer's instructions. RNA quality was examined using an Agilent 2100 Bioanalyzer. Total RNA from the same experimental group was pooled prior to the construction of the small RNA library.

### Small RNA library construction and sequencing

Small RNA fragments (18–30 nt) were isolated from total RNA using a Novex 15% TBE-Urea gel (Life Technologies). Then, a 5′-adaptor (Illumina, San Diego, CA, USA) was ligated to the small RNAs, and the products were purified on a Novex 15% TBE-Urea gel to remove any non-ligated adaptors. The 5′ ligation products (36–50 nt) were then ligated to a 3′-adaptor (Illumina) and purified on a Novex 10% TBE-Urea gel (Life Technologies). Ligation products with adaptors at both ends (62–75 nt) were then reverse-transcribed and PCR-amplified using adaptor primers. The amplification products were excised from a 6% TBE-Urea gel (Life Technologies). The purified cDNA library was used for clustering and sequencing analysis using a HiSeq 2000 Illumina sequencer at the Beijing Genomics Institute (BGI), Shenzhen, China.

### Data analysis

Sequencing data were uploaded to the NIH Short Read Archive (project accession NO. SRP039387). Raw data from the HiSeq sequencing were first filtered and cleaned. The low-quality reads, including reads with no 3′ adapter, reads with no insertion, reads with 5′ adapter, reads smaller than 18 nt, and reads with a polyA tail, were removed. The length distribution of the clean tags was then summarized. The clean reads were then mapped to miRBase19 (http://www.microrna.org/) and the *T. nigroviridis* genome to identify the conserved miRNAs. The small RNA reads were also aligned to repeat associated RNA, exons and introns of mRNA, rRNA, scRNA, snoRNA, snRNA, and tRNA. The small RNA tags were then annotated using the software tag2annotation developed by BGI.

### Identification of differentially expressed miRNAs and target prediction

The miRNA expression profiles of the control and rIFN-γ-treated groups were compared to identify differentially expressed miRNAs. The expression of the miRNAs in the two samples (control and treatment) was normalized to determine the expression as transcripts per million (TPM). Then, the fold change and P-value were calculated from the normalized expression, and a log2-ratio scatter plot was generated. MiRNAs with similar expression patterns were clustered using hierarchical clustering, as previously described [51].

The targets of the annotated miRNAs were predicted using Mireap software developed by BGI. The rules used for target prediction were based on previously described suggestions [52], [53]. KOG analysis was performed to classify the targets by their functions. The top three targets with the highest scores among the differentially expressed miRNAs were analyzed using GO enrichment and KEGG pathway analysis.

### Reverse transcription and quantitative polymerase chain reaction (RT-qPCR)

*T. nigroviridis* miRNA expression levels were measured as previously described [54]. RNA samples that were used in the HiSeq sequencing analysis were reverse-transcribed and amplified using the Hairpin-it miRNAs RT-PCR Quantitation kit (GenePharma, Shanghai, China). The primers used in the reverse transcription and real-time PCR reactions were provided by GenePharma (Shanghai, China). Real-time quantitative PCR was performed on an ABI 7900HT instrument. The reactions were incubated at 95°C for 3 min, followed by 40 cycles of 95°C for 12 sec and 62°C for 40 sec. All reactions were run in triplicate. *T. nigrovir*idis U6 snRNA was used as a control. Relative miRNA expression was calculated using the comparative threshold (2^-ΔΔCt^) method [48]. The Ct values used in the calculation were the means of the triplicates, and the data are presented as means ± SEM. Significant differences were analyzed using t-tests, and p<0.05 was considered statistically significant.

## Results

### High-throughput sequencing of small RNAs

To identify differentially expressed miRNAs after rIFN-γ treatment, spleen cells from *T. nigroviridis* were divided into three groups: the control group (Sp-con), the rIFN-γ1-treated group (Sp-γ1), and the rIFN-γ2-treated group (Sp-γ2). All three groups were sequenced separately. In total, 11,899,197 raw reads were obtained from the Sp-con group, whereas 12,000,000 raw reads were obtained from both the Sp-γ1 and Sp-γ2 groups. After the low-quality reads were removed, 11,661,792, 11,821,415, and 11,705,803 clean reads were obtained from the Sp-con, Sp-γ1, and Sp-γ2 groups, respectively. The length distributions of the three groups were analyzed (Figure 1); the reads were mainly 22–23 nt in length, similar to previous studies [14], [55], [56]. The clean reads were then mapped to the mature miRNAs of all animals in miRBase19, as only 132 *T. nigroviridis* miRNA records could be found in miRBase19. In total, 1556, 1538, and 1573 mature miRNA sequences were identified in the Sp-con, Sp-γ1, and Sp-γ2 groups, respectively. All miRNAs were mapped to the *T. nigroviridis* genome (Figure 2). All of the identified miRNA sequences are listed in Supplemental Table S1.

**Figure 1:** Read length distribution of the clean reads from the (A) Sp-con, (B) Sp-γ1, and (C) SP-γ2 groups.

**Figure 2:** Small RNA tags matched to the genome by SOAP. The figure shows the expression and genomic distribution of miRNAs identified in the (A) Sp-con, (B) Sp-γ1, (C) SP-γ2 groups.

### Identification of differentially expressed miRNAs

The known miRNA reads were compared between the Sp-con/Sp-γ1, Sp-con/Sp-γ2, and Sp-γ1/Sp-γ2 groups to identify the differentially expressed miRNAs. The log2 ratio and p-value were calculated, and miRNAs with a log2 ratio >1 and p<0.05 were considered to be up-regulated; miRNAs with a log2 ratio <−1 and p<0.05 were considered to be down-regulated. The miRNAs differentially expressed among different experiment groups were summarized using hierarchical clustering (Figure 3) and the log2-ratio scatter plot (Figure 4). The above analyses indicate that 191 miRNAs were significantly up-regulated and that 207 miRNAs were significantly down-regulated after rIFN-γ1 stimulation; after rIFN-γ2 stimulation, 226 miRNAs were significantly up-regulated and 212 miRNAs were significantly down regulated. In total, 403 miRNAs were differentially expressed between the two groups treated with rIFN-γ1 and rIFN-γ2 (Supplemental Table S2). qRT-PCR was used to verify the expression profile of the differentially expressed miRNAs. In total, 10 differentially expressed miRNAs (tni-miR-106a-3p, tni-miR-124b-3p, tni-miR-132-3p, tni-miR-142-3p, tni-miR-145b, tni-miR-17, tni-miR-223-5p, tni-miR-29d-3p, tni-miR-346, and tni-miR-378) were selected for PCR validation. The normalized read counts of the 10 selected miRNAs are shown in Figure 5. Whereas tni-miR-124b-3p and tni-miR-17 were differentially expressed after both rIFN-γ1 and rIFN-γ2 treatment, the other eight miRNAs were differentially expressed only after either rIFN-γ1 or rIFN-γ2 treatment. The real-time PCR validation of these 10 miRNAs is shown in Figure 6. All of the 10 selected miRNAs showed the same pattern of increase or decrease suggested by the sequencing data, although the magnitude of the change in tni-miR-106a-3p, tni-miR-17, and tni-miR-346 expression was different between the sequencing results and PCR data.

**Figure 3:** Expression of the identified miRNAs in the three different samples using hierarchical clustering. Highly expressed miRNAs are indicated in red, and miRNAs with low expression are indicated in green; grey indicates missing data. The absolute signal intensity ranged from −4.0 to +4.0.

**Figure 4:** Log2-ratio scatter plot of the differentially expressed miRNAs between (A) the Sp-con and Sp-γ1 groups, (B) the Sp-con and Sp-γ2 groups, and (C) the Sp-γ1 and SP-γ2 groups. Each point in the figure represents a miRNA. The X and Y axes show the expression levels in the two samples. The red points represent miRNAs with a ratio >2, the blue points represent miRNAs with a ratio >1/2 and ≤2, and the green points represent miRNAs with a ratio ≤1/2.

**Figure 5:** Normalized read counts for selected miRNAs. (A): Normalized read counts for miR-124b-3p, miR-142-3p, miR-145b, miR-17, miR-29d-3p, and miR-346 following IFNγ1 treatment, compared to the control group. (B): Normalized read counts of miR-106a-3p, miR-124b-3p, miR-132-3p, miR-17, miR-223-5p, and miR-378 following IFNγ2 treatment, compared to the control group.

**Figure 6:** Quantitative real-time PCR validation of selected miRNAs. (A): expression of miR-124b-3p, miR-142-3p, miR-145b, miR-17, miR-29d-3p, and miR-346 following IFNγ1 treatment, compared to the control group. (B): expression of miR-106a-3p, miR-124b-3p, miR-132-3p, miR-17, miR-223-5p, and miR-378 following IFNγ2 treatment, compared to the control group. The amount of each miRNA was normalized to that of U6 snRNA and is presented as the relative fold change (n = 3, mean ± SEM). Significant differences between the control and treatment groups are indicated (*P<0.05; **P<0.01; ***P<0.001).

### Target prediction

The *T. nigroviridis* genome database was used to predict miRNA targets. In total, 165,369 genes were predicted to be targets of expressed miRNAs, and these genes were annotated in the KOG database and divided into 25 groups (Figure 7). Among these 25 groups, genes involved in signal transduction mechanisms were the most commonly targeted genes (13.83%), followed by genes involved in translation, ribosomal structure and biogenesis (12.69%) and those involved in the cytoskeleton (11.08%).

**Figure 7:** KOG classes of predicted targets for *Tetraodon nigroviridis* miRNAs.

To further investigate the differentially expressed miRNAs, the top three targets with the highest scores among all the differentially expressed miRNAs were analyzed using GO and KEGG analyses (Supplemental Table S3–S6). The results showed that many target genes were deeply involved in the IFN-γ-mediated immune response. For example, SOCS3 (GenBank accession NO. CR675748), GALT (CR677385), CRFA22 (AY374494), CISH (EF195753), and CRFA28 (CR734177) are involved in the Jak-Stat signaling pathway, whereas BPI (CR648786), SYNGR2 (CR663898), CRFB3 (CR726689, CR733157) are involved in the Toll-like receptor signaling pathway. NLRC3 (CR655744), HSP90AA (CR646339), and IAP (CR709695) are involved in the NOD-like receptor signaling pathway, and MHC I (CR635680), IgL-3 (AJ575617), calreticulin (CR639214), and CD4-2 (CR733985) are involved in antigen processing and presentation. The predicted targets for the differentially expressed miRNAs are summarized in Supplemental Table S7. The target prediction for the differentially expressed miRNAs and the functions of the predicted targets require further investigation.

## Discussion

MiRNAs have been shown to be involved in the innate and acquired immune response [57], [58]. Using high-throughput sequencing technology, we were able to identify differentially expressed miRNAs in *T. nigroviridis* spleen cells after stimulation with recombinant IFN-γs. IFN-γ is critically involved in innate and adaptive immunity, and is an important activator of macrophages. IFN-γ has been studied in teleosts [59], as two copies of the IFN-γ gene have been found in many fish species [35], [36], [60], thus raising interest in the teleost IFN-γ system. *T. nigroviridis* has the smallest known vertebrate genome; however, few studies concerning *T. nigroviridis* miRNAs have been reported [61]. Our group previously identified two IFN-γ genes in *T. nigroviridis*, and our present study has identified miRNAs involved in the response to two IFN-γs. To our knowledge, this is the first study to investigate IFN-γ-related miRNAs in teleosts.

Using Solexa high-throughput sequencing, we identified 1556, 1538, and 1573 mature miRNA sequences in the SP-con, SP-γ1 and SP-γ2 samples, respectively. All of the identified miRNAs were mapped to miRBase19 to identify the conserved miRNAs. Because only 132 miRNA records for *T. nigroviridis* were found in miRBase19, we mapped the sequencing reads to miRNAs of all animals in miRBase. We identified many *T. nigroviridis* miRNAs that were not recorded in miRBase, such as miR-764-5p (5′-GGUGCCCGCAUCCUCCUCCA-3′), miR-346 (5′- TGTTGCCCGCATCCTCCAC-3′), and miR-146a-5p (5′-TGAGAACTGAATTCCATCGCTGGTT-3′). All of the identified *T. nigroviridis* miRNAs are listed in Supplemental Table S1. Among these miRNAs, 397 miRNAs were differentially expressed between the control and IFN-γ1 groups, and 438 miRNAs were differentially expressed between the control and IFN-γ2 groups; additionally, 403 miRNAs were differentially expressed between the two IFN-γ treatment groups (Supplemental Table S2). Different miRNA expression patterns were observed after rIFN-γ1 and rIFN-γ2 treatment, suggesting that both IFN-γ1 and IFN-γ2 may be functional and may regulate the *T. nigroviridis* immune system. Next, we verified the differential expression data using qRT-PCR. Ten miRNAs were selected for verification, including tni-miR-106a-3p, tni-miR-124b-3p, tni-miR-132-3p, tni-miR-142-3p, tni-miR-145b, tni-miR-17, tni-miR-223-5p, tni-miR-29d-3p, tni-miR-346, and tni-miR-378. The qPCR results showed the same up- and down-regulation patterns indicated by the sequencing data. Previous studies concerning the identified differentially expressed miRNAs showed that these miRNAs are involved in many immunological progresses in other species or cell lines.

First, we focused on previous studies of miR-106a-3p, miR-17 and miR-124b-3p in mammals. MiR-106a-3p, which belongs to the miR-17 family, is involved in many types of tumors [62], [63], [64]; additionally, miR-106a directly regulates Stat3 [65] and IL-10 [66]. Stat3 is the signal transducer for IFN-γ in some cell types [23], whereas IL-10 inhibits IFN-γ production through inhibition of IL-12 [67], [68]. MiR-17 is a member in the miR-17∼92 cluster and acts as a potential oncogene [69]. In addition to its oncomiR function [70], [71], miR-17 regulates macrophage differentiation [72] and macrophage inflammatory responses [73] and is also involved in Stat3 signaling [74]. Both miR-106a and miR-17 are regulated by c-Myc [75], [76], which is a transcription factor that can be suppressed by IFN-γ [77]. MiR-124b-3p belongs to the miR-124 family, and tni-miR-124b-3p is highly conserved with human miR-124 (100% identity to the mature sequence), which has been demonstrated to target Stat3 in different types of cancer [78], [79], [80]. These studies indicate that miR-106a-3p, miR-17, and miR-124b-3p may be involved in Stat3-dependent IFN-γ signaling. MiR-106a-3p may also be involved in feedback control of IFN-γ expression by targeting IL-10, and miR-17 may also participate in the IFN-γ-mediated activation of macrophages.

We next focused on miRNAs relevant to IFN-γ-induced cytokines. IL-12 is induced by IFN-γ and then up-regulates IFN-γ through a feedback mechanism [81]. It has been reported that miR-132-3p is up-regulated after IL-12 treatment, and this up-regulation decreases Stat4 and IFN-γ expression [82]. MiR-142-3p, a hematopoietic-specific miRNA [83], was down-regulated after rIFN-γ1 treatment in our study, and previous studies have shown that down-regulation of miR-142-3p can increase IL-6 expression [84], resulting in CD4^+^ T cell activation [85] and macrophage differentiation in tumors [86]. IL-6 is a proinflammatory cytokine whose production can be activated by the LPS-induced macrophage response, and IFN-γ is known to prime macrophages to enhance their response to LPS [87], [88]. Additionally, IFN-γ primes helper T cell differentiation and macrophage differentiation [89]. The suppression of miR-142-3p indicates a synergistic effect of miR-142-3p and IFN-γ in the priming of macrophage responses. MiR-223-5p is the passenger strand of miR-223; although few studies about the passenger strand have been published, a decrease in miR-223 inhibits LPS-induced IFN-γ production in splenic lymphocytes [90]. Additionally, down-regulation of miR-223 resulted in the activation of Stat3 and promoted the production of Toll-like-receptor (TLR)-triggered IL-6 and IL-1β [91], indicating that miR-223-5p may function in the IFN-γ priming of the LPS response and Stat3-dependent IFN-γ signaling. Finally, although only a few studies of miR-346 have been undertaken, some reports have linked miR-346 to the immune system because of its ability to control the release of IL-18 and TNFα, and its targeting of TAP1 [92], [93], [94]. These studies suggest that miR-346 may also be involved in the priming of the LPS response.

Another down-regulated miRNA, tni-miR-145b, is highly similar to human miR-145 (94.7% identical with one mismatch in the 3' end). Studies have shown that miR-145 expression is also decreased in various human tumors [95], [96]. Additionally, in cancer cells, miR-145 is reported to target Stat1 [47], the main signal transducer of the IFN-γ pathway, in addition to c-Myc [46], [97]. Recent studies have also revealed that miR-145 regulates IFN-β expression by targeting the suppressor of cytokine signaling (SOCS)7 [98]. These data indicate that miR-145 may regulate the major IFN-γ signaling pathway and may also participate in crosstalk among other interferons. Another miRNA, tni-miR-29d-3p, belongs to the miR-29 family and has 95.4% identity (one mismatch in the 3′ end) with human miR-29b. The miR-29 family has been shown to directly target IFN-γ [44], [99], and IFN-γ-induced Stat1 could control miR-29 expression through a feedback mechanism [45], suggesting that miR-29d-3p may be a crucial factor in the IFN-γ-mediated immune responses that control the production of IFN-γ itself. Previous studies have also shown that miR-378 can target the IFN-γ receptor gene IFNGR1 and suppress bovine luteal cell apoptosis [48]. These findings indicate that these differentially expressed miRNAs may play crucial roles in the IFN-γ-mediated immune response, and the interactions between these miRNAs and IFN-γ should be researched further.

Additionally, seven out of the 10 validated miRNAs (miR-124b-3p, miR-132-3p, miR-142-3p, miR-145b, miR-17, miR-29d-3p, and miR-346) were differentially expressed between the IFN-γ1 and IFN-γ2 treatment groups, suggesting functional segregation or synergy of the two fish IFN-γ isoforms. Previous studies on the two fish IFN-γ isoforms showed that they bind to different receptors and exhibit different expression patterns [36], [40], [41]. Comparative studies on the two IFN-γ isoforms showed that they have complementary and also overlapping functions [39], [40], [41]. The miRNA differential expression data also suggest that the two isoforms have separate functions; for example, miR-124b-3p and miR-17 were down-regulated after rIFN-γ1 treatment but were significantly up-regulated after rIFN-γ2 treatment. As mentioned above, miR-124b-3p and miR-17 may be involved in Stat3-dependent IFN-γ signaling, which suggests that IFN-γ1 and IFN-γ2 may have opposite effects on the Stat3 signaling pathway in *T. nigroviridis*. Previous studies in mammals have indicated that miR-106a and miR-17 were up-regulated after 12 h of IFN-γ treatment [100], which is in agreement with our findings for IFN-γ2, suggesting that *T. nigroviridis* IFN-γ2 may be closely related to mammalian IFN-γ. Additionally, the rIFN-γ1-specific down-regulation of miR-145b indicates that IFN-γ1 may be involved in the Stat1-dependent signaling, and the rIFN-γ1-specific up-regulation of miR-29d-3p suggests that IFN-γ1 may participate in the feedback control of IFN-γ. Furthermore, the rIFN-γ2-specific induction of miR-132-3p indicates that IFN-γ2 may be responsible for IL-12 production. The differential expression of miRNAs between the two treatment groups may provide important information regarding the functional segregation of the two fish type II IFN isoforms.

The targets of all the *T. nigroviridis* miRNAs were predicted using Mireap software, and KOG analysis was performed. The KOG results showed that most of the target genes function in signal transduction mechanisms; translation, ribosomal structure, and biogenesis; and the cytoskeleton. Most of the target genes that function in signal transduction were also found in previous miRNA high-throughput sequencing studies [15], [56]. To determine the function of the differentially expressed miRNAs, their targets were predicted. Because the results of the target prediction were redundant, we chose only the top three targets with the highest scores for further analysis (Supplemental Table S7). These filtered targets were analyzed using GO enrichment and KEGG pathway analysis, and from the GO and KEGG analyses, we assembled a model of the miRNA-protein interaction network; however, the actual system may be much more complicated and may require further study for elucidation. Some target genes were predicted to be involved in components of the IFN-γ-mediated immune response, such as the Jak-Stat signaling pathway, the Toll-like receptor signaling pathway, the NOD-like receptor signaling pathway, the T cell receptor signaling pathway, antigen processing and presentation, and natural killer cell-mediated cytotoxicity. Targets involved in these pathways should be evaluated in future studies concerning IFN-γ-induced miRNAs. However, computational methods for miRNA target prediction often have false positive rates [101], [102]; thus, further analysis is needed to confirm the interaction between miRNAs and their targets.

In conclusion, using high-throughput sequencing technology, we studied the *T. nigroviridis* miRNAs expressed in spleen cells. Many miRNAs were identified after rIFN-γ1 and rIFN-γ2 stimulation of spleen cells, and differentially expressed miRNAs were identified and validated using qRT-PCR. The miRNA targets were predicted and analyzed using GO and KEGG analyses. This study provides the basis for the interaction between *T. nigroviridis* IFN-γ and miRNAs, and these data provide clues for further studies on the mechanisms of IFN-γ-mediated immune responses in *T. nigroviridi*s.

## Supporting Information

Table S1 **All mature miRNA sequences identified using Solexa high-throughput sequencing.**
(XLS)

Table S2 **MiRNAs differentially expressed between the control and IFNγ1/IFNγ2-treated groups.**
(XLS)

Table S3 **GO enrichment analysis of the predicted mRNA targets of the miRNAs differentially expressed between the SP-con and Sp-γ1 groups.**
(XLS)

Table S4 **GO enrichment analysis of the predicted mRNA targets of the miRNAs differentially expressed between the Sp-con and Sp-γ2 groups.**
(XLS)

Table S5 **GO enrichment analysis of the predicted mRNA targets of the miRNAs differentially expressed between the Sp-γ1 and Sp-γ2 groups.**
(XLS)

Table S6 **KEGG pathway analysis of the predicted mRNA targets of the differentially expressed miRNAs.**
(XLS)

Table S7 **Predicted mRNA targets of the differentially expressed miRNAs.**
(XLS)
